# Analysis of Risk Factors for Postoperative Lower Extremity Deep Venous Thrombosis and its Treatment and Nursing

**DOI:** 10.1155/2022/9180696

**Published:** 2022-09-08

**Authors:** Huayun Liu, Yunhua Peng

**Affiliations:** ^1^The Affiliated Nanhua Hospital,Department of Gastroenterology, Hengyang Medical College, University of South China, Hengyang, Hunan 421001, China; ^2^The Affiliated Nanhua Hospital,Department of Spine Surgery, Hengyang Medical College, University of South China, Hengyang, Hunan 421001, China

## Abstract

**Objective:**

To explore the risk factors of lower extremity deep venous thrombosis (LEDVT) after surgery and discuss the treatment and nursing countermeasures.

**Methods:**

A retrospective analysis was conducted on 268 surgical patients admitted between July to December 2021. The factors associated with LEDVT were analyzed using the Logistic regression model. Further, LEDVT patients were assigned to a research group treated with targeted nursing to prevent LEDVT and a control group that used routine care. Coagulation function and inflammatory cytokines before and after nursing intervention were compared between groups. The assessment of patients' mobility employed the lower limb motor function part of the Fugel–Meyer Assessment (FMA), Harris Hip Score (HHS), and Barthel index (BI), and their psychological status was evaluated using the Kolcaba's General Comfort Questionnaire (GCQ) and Self-rating Anxiety/Depression Scale (SAS/SDS). Finally, patient satisfaction with the treatment service was investigated.

**Results:**

Logistic regression analysis showed that hypertension, limb paralysis, central venous catheterization of lower limbs, and bedridden time affect postoperative LEDVT in an independent way (*P* < 0.05). After the intervention, the coagulation function and inflammatory reaction were improved in both groups, with more significant improvement in the research group (*P* < 0.05). The research group also showed higher FMA, Harris, GCQ, and BI scores while lower SAS and SDS scores than the control group postnursing intervention (*P* < 0.05). Finally, a higher satisfaction rate was identified in the research group as compared to the control group (*P* < 0.05).

**Conclusion:**

Hypertension, limb paralysis, CVC of lower limbs, and bedridden time are all independent risk factors for LEDVT after surgery. The implementation of targeted nursing strategies for the above factors can effectively alleviate the hypercoagulable state of patients after operation, reduce inflammatory responses, and improve patient comfort, which is of great significance for preventing the occurrence of LEDVT.

## 1. Introduction

Surgery, an important treatment modality in clinical practice, is the only resort for multiple diseases. According to statistics, an average of 2–6 surgical operations are performed every day in grade III-A hospitals [1]. However, this mechanically invasive procedure may negatively affect patients to varying degrees and lead to postoperative complications [2]. Among them, lower extremity deep venous thrombosis (LEDVT) is a very common complication after surgical operation, mainly attributed to reduced physical activity due to limited range of motion, weakened muscle pump, and vascular obstruction caused by invasive procedures [3]. Studies have shown that more than 40% of surgical patients may have LEDVT after surgery, and the incidence rate of LEDVTis increasing year by year [4]. LEDVT may not only have a great negative impact on patients' postoperative rehabilitation but also cause blood supply disorders, resulting in organ dysfunction and disorders, and even sudden cardiac death in severe cases [5]. Because of this, LEDVT has become the focus of medical workers at home and abroad, and how to effectively prevent and control the occurrence of LEDVT has become a hot spot of modern medical research [6].

As the first line of defense against LEDVT, risk assessment plays a vital part in clinical practice [7]. LEDVT prevention programs for general surgical patients based on accurate risk assessments can minimize the incidence of the LEDVT. However, in clinical practice, nursing staff still lack understanding of the LEDVT risk factor identification, the timing ofLEDVT risk assessment, and the correct use of the LEDVT risk assessment scales [8]. Coupled with a lack of authoritative unified clinical guidelines, all of which leads to inaccurate identification and risk stratification of the LEDVT risk factors in general surgical patients, as well as the negative prevention or excessive prevention is common, greatly affecting the perioperative rehabilitation of patients and the identification of potential risk of the LEDVT [9]. Therefore, an in-depth understanding of the risk factors for LEDVT occurrence, early identification, and accurate risk assessment are of great significance for the prevention and control of LEDVT in patients.

Based on the above-given theory, this study analyzes the risk factors of postoperative LEDVT and discussed the treatment and nursing countermeasures, so as to provide reliable and accurate reference and guidance for future clinical prevention and treatment of the LEDVT.

## 2. Materials and Methods

### 2.1. Patient Data

A retrospective analysis was conducted on 268 surgical patients admitted between July to December 2021. Among all the patients, 79 patients developed LEDVT after surgery, of which 36 patients received LEDVT targeted care and were regarded as the research group (RG), and 43 patients received routine post-operative care and were assigned to the control group (CG). This study strictly followed the Declaration of Helsinki, and all subjects signed informed consent.

Diagnostic criteria of LEDVT: ① the clinical manifestations are sudden limb pain, swelling, and increased soft tissue tension; ② the plasma D-D level is above 500 *μ*g/L; ③ the diagnosis is confirmed by Doppler ultrasonography and venography.

### 2.2. Eligibility Criteria

The enrolled patients (age >18 years) all underwent surgical treatment in our hospital and agreed to participate in this research, with complete medical records. Those meeting any of the following criteria were excluded: blood dysfunction; vascular occlusive diseases; long-term coma without self-consciousness; pregnant and lactating patients; organ dysfunction or disorders; referred patient.2.

### 2.3. Methods

Routine nursing: nursing staff closely monitor the patient's condition, educate the patient about health knowledge to prevent postoperative complications, and regularly turn the patient over to prevent pressure ulcers. The nursing staff closely monitored the patient's condition, gave the patient health knowledge and education on the prevention of postoperative complications, and regularly turned over the patient to prevent pressure ulcers. Nursing for LEDVT: a LEDVT nursing team was established, with a senior director-level nurse serving as the team leader, and the team members were trained on LEDVT prevention. The nursing staff in the group could only start the practice after passing the theoretical and operational skills assessment. The risk assessment of patients was carried out, the risk factors of LEDVT were summarized, judging whether there are risk factors in patients, and the targeted measures were given. The seriousness and harm of post-operative LEDVT, as well as routine prevention and treatment, were explained to patients and their families by means of health brochures, video broadcasts, in-hospital expert lectures, etc., so as to inform them of the importance of actively cooperating with treatment and enhance their cognition of LEDVT and treatment compliance. For postural nursing, patients were required to raise their feet by 20°–30°, and hot compress and massage were performed on both lower limbs regularly. In addition, they were helped to turn over every 2 hours and encouraged to ambulate as soon as possible, exercise the lower limbs and change their postures more frequently. Patients were also accompanied by nursing staff or family members for indoor walking training, twice a day, with each walking time not exceeding 30 min. Those who were not suitable to get out of bed were instructed to raise their lower limbs, do passive exercises such as flexion and extension and varus-valgus of joints and lower limbs, and massage. Elastic bandages, elastic socks, and air pressure therapy were also given as appropriate. Furthermore, assess the patient's psychological state, provide timely psychological counseling, answer the patient's questions earnestly and eliminate the patient's confusion. Communication with patients and their families was strengthened, and nursing staff helped eliminate patients' negative emotions through encouraging language, music, meditation and relaxation training. More importantly, the patient's dietary regimen was reasonably formulated to prevent platelet aggregation and recurrence of LEDVT. During the intervention period, the team leader and clinicians regularly spot check the work within the team, timely find and solve problems, and constantly summarize and improve the quality of clinical nursing management and service.

### 2.4. Sample Collection and Testing

Before and after the nursing intervention, fasting peripheral blood was sampled and divided into two parts. One part was tested by an automatic coagulation function analyzer for prothrombin time (PT), activated partial thromboplastin time (APTT), plasma thrombin time (TT), fibrinogen (FIB), and D-dimer (D-D). The other part was used for the determination of high-sensitivity C-reactive protein (hs-CRP), procalcitonin (PCT), and tumor necrosis factor-*α* (TNF-*α*) by ELISA after centrifugation for 30 min to obtain serum.

### 2.5. Evaluation Criteria

The lower limb motor function part of the Fugel–Meyer Assessment (FMA) scale, Harris Hip Score (HHS), and Barthel index (BI) were used to evaluate the lower limb motor function of the patient, with a total score of 34 points, 100 points, and 100 points, respectively. The score of each scale is in direct proportion to the motor function. Patient comfort (Kolcaba's General Comfort Questionnaire, GCQ) and psychological states (Self-Rating Anxiety/Depression Scale [SAS/SDS]) were also evaluated. The total score of GCQ is 28–112 points, and the score is positively related to the comfort level. For SAS and SDS, the score is converted by multiplying the score by 1.25, with a total score of 0–100 points. Higher scores suggest more serious anxiety and depression. An anonymous satisfaction survey was conducted upon the discharge of patients. According to the score, the satisfaction was divided into very satisfied (>80 points), basically satisfied (60–80 points), or dissatisfied (<60 points). Total satisfaction rate = (very satisfied + basically satisfied)cases/total cases × 100%.

### 2.6. Endpoints

(1) The related factors affecting the occurrence of LEDVT after surgery were analyzed; (2) alterations of coagulation function, inflammatory cytokines (ICs), mobility, and psychological states were recorded before and after the nursing intervention; (3) patients' satisfaction with treatment services was investigated at discharge.

### 2.7. Statistical Methods

Data were statistically analyzed by SPSS22.0, and differences with *P* < 0.05 were considered significant in this study. A Chi-square test was used for intergroup comparison of count data expressed as (%) or [n (%)]. For measurement data recorded in the form of (‾*χ*±*s*), the intergroup and within-group differences were identified by independent sample *t*-test and paired *t*-test, respectively. Relative risk factors were analyzed using the Logistic regression model.

## 3. Results

### 3.1. Univariate Analysis of Factors Influencing the Occurrence of LEDVT

First, 268 patients were assigned to either the DVT group (*n* = 79) or the non-DVT group (*n* = 189) according to the occurrence of LEDVT, followed by a univariate analysis. As shown in Table 1, the two groups showed no statistical difference in sex, disease type, and operation type (*P* > 0.05), which indicated that none of the above indexes was a single factor affecting the occurrence of LEDVT. However, the DVT group had higher age, BMI, hypertension, limb paralysis, central venous catheterization (CVC) of lower limbs, and bedridden time than the non-DVT group (*P* < 0.05), suggesting that these indicators were single factors affecting the occurrence of LEDVT.

### 3.2. Multivariate Analysis of Factors Affecting the Occurrence of LEDVT

After assigning the above-mentioned indicators with differences (Table 2) and inputting them into SPSS, Logistic regression analysis was carried out with whetherLEDVT occurred or not as an independent variable and other indexes as covariates. The output results showed that age and BMI were not independent factors for postoperative LEDVT (*P* > 0.05), but hypertension, limb paralysis, CVC of lower limbs and bedridden time were (*P* < 0.05; Table 3).

### 3.3. Comparison of Coagulation Function before and after Nursing Intervention

The coagulation function parameters TT, PT, APTT, FIB, and D-D were not statistically different between groups before intervention (*P* > 0.05). TT, PT, and APTT elevated notably in both cohorts after the intervention and were higher in RG compared with CG (*P* < 0.05); while obvious decreases in FIB and D-D were observed in both cohorts, with lower values in RG (*P* < 0.05; Figure 1).

### 3.4. Comparison of ICs before and after Intervention

The test results of ICs showed no evident differences in hs-CRP, PCT, and TNF-*α* between groups before intervention (*P* > 0.05). But the levels of these ICs reduced markedly in both cohorts, especially in RG (*P* < 0.05; Figure 2).

### 3.5. Comparison of Mobility before and after Intervention

The FMA, HHS, and BI scores were found to be similar in the two groups before intervention (*P* > 0.05). However, all the three scores elevated remarkably after intervention (*P* < 0.05), with more obvious increases in RG (*P* < 0.05; Figure 3).

### 3.6. Comparison of Psychological States before and after Intervention

GCQ, SAS, and SDS scores differed insignificantly between the two groups before intervention (*P* > 0.05). After the intervention, the GCQ score increased and the SAS and SDS scores decreased in both cohorts (*P* < 0.05), and the increase in GCQ score and decreases in SAS and SDS scores were more significant in RG (*P* < 0.05; Figure 4).

### 3.7. Comparison of Satisfaction

The satisfaction survey results are shown in Table 4. 66.67% of patients in RG were very satisfied with the intervention, and 34.88% of patients in CG. The overall satisfaction rate in RG was 94.44%, a rate higher than that of 79.07% in CG (*P* < 0.05).

## 4. Discussion

LEDVT, as one of the most commonly seen postoperative complications, has an increasing incidence in recent years with the popularity of surgery [10]. At present, although there are some clinical studies on the prevention and treatment of LEDVT [11–13], the results are not completely consistent, and there is still great controversy about the postoperative response measures. In this study, significant and excellent results have been achieved in the prevention of postoperative LEDVT through analyzing the related factors and implementing targeted prevention and care strategies. Hence, this research has important reference significance for the followup clinical research and the formulation of LEDVT prevention and treatment strategies.

We first analyzed factors associated with postoperative LEDVT. The results showed that hypertension, limb paralysis, CVC of lower limbs, and bedridden time were all independent risk factors for LEDVT after surgery. First of all, it is well known that hypertension, as a very common underlying chronic disease, has more than 100 million cases worldwide [14]. The presence of hypertension can make the blood circulation in the patient's body in a long-term high pressure state, which leads to the generation of internal shear force of the blood vessel wall, resulting in vascular stenosis and sclerosis, and eventually thrombosis [15, 16]. Therefore, the possibility of LEDVT would be significantly increased in hypertensive patients, which is consistent with previous research results and supports our results [17, 18]. On the other hand, patients with paralysis are naturally at increased risk of LEDVT because their mobility is completely lost. Similarly, the findings of Desmukh's team also suggest that limb paralysis is a risk factor for LEDVT [19]. Lower extremity CVC is a mechanical invasive procedure, which has been repeatedly confirmed to cause LEDVT [20, 21] and is related to the destruction of intravascular stability and the increased risk of infection. Finally, for the bedridden time, it is also associated with the reduction of limb mobility and muscle pump as described above, thus also contributing to an increased risk of LEDVT. Based on the above results, we believe that the core of LEDVT prevention and treatment includes the following three points: (1) focusing on the relief of basic chronic vascular diseases; (2) strengthening patients' post-operative activities, and enhancing muscle pumps; (3) avoiding mechanical invasive procedures as much as possible.

Then, in view of the above conclusions, we formulated nursing strategies for preventing and treating postsurgical LEDVT and put them into clinical use. The evaluation results showed that RG receiving targeted nursing had higher TT, PT, and APTT than CG treated by conventional nursing, with lower FIB, D-D, hs-CRP, PCT, and TNF-*α* levels. The results showed that the coagulation function in RG was better and the inflammation in RG was less after the nursing intervention, which indicated that the targeted nursing implemented in this study could effectively alleviate the hypercoagulable blood state and inflammatory reaction injury of patients after surgery, and promote the postoperative rehabilitation of patients. Due to the lack of activity of the lower limbs caused by long-term bedridden, the blood flow slowed down and stagnated, and the blood showed a hypercoagulable blood state [22]. At the same time, due to the mechanical operation, the inflammatory injury reaction in the body is intensified [23]. While increasing the mobility of patients' limbs through active posture nursing, massage, and activity guidance, the targeted nursing developed in this study can promote blood circulation and reduce blood hypercoagulability and inflammation, thus preventing thrombosis. In addition, the nursing strategy provides patients and their families with comprehensive health education, standardized postural care, and early preventive nursing intervention, so that patients and their families can learn more about postoperative recovery and LEDVT, improve patient compliance and ensure that patients are always in a scientific posture after surgery. The risk factors of venous thromboembolism can be reduced by the scientific functional exercise of the affected limb. This can also be confirmed by the physical mobility scores of the two groups. Moreover, after nursing, the GCQ score of RG increased, and the SAS and SDS scores of RG decreased, which also indicated that the nursing strategy could mitigate patients' bad mood and enhance their physical comfort. The main reason is that the nursing project pays attention to the psychological state of patients, which helps patients to solve their own psychological problems, adjust their psychological state, and alleviated the patients' bad mood caused by their illness. At the same time, reasonable nursing strategies can alleviate the symptoms of physical discomfort such as limb pain and itching, improve the patient's physical comfort, and further reduce the adverse effects of physical discomfort on patients' psychology and quality of life. Finally, the improvement in the treatment satisfaction of RG again verified the success of this strategy, indicating that it is worthy of future clinical promotion.

However, there are still many limitations to be improved in this research. Because of the short experimental period, we are unable to evaluate the long-term prognosis of patients for the time being. And, due to the lack of clinical guidelines, the nursing strategy to prevent LEDVT needs to be continuously improved and optimized. Finally, we need to expand the number of cases to obtain more representative results, in order to provide a reference for clinical practice.

In conclusion, hypertension, limb paralysis, CVC of lower limbs, and bedridden time are all independent risk factors for LEDVT after surgery. The implementation of targeted nursing strategies for the above factors can effectively alleviate the hypercoagulable state of patients after operation, reduce inflammatory responses, and improve patient comfort, which is of great significance for preventing the occurrence of LEDVT.

## Figures and Tables

**Figure 1:** Comparison of coagulation function before and after the nursing intervention. (a) TT comparison between the two groups. (b) PT comparison between the two groups. (c) APTT comparison between the two groups. (d) FIB comparison between the two groups. (e) D-D comparison between the two groups. ^#^means comparison with before intervention (*P* < 0.05), ^&^means comparison with RG (*P* < 0.05).

**Figure 2:** Comparison of ICs before and after an intervention. (a) hs-CRP comparison between the two groups. (b) PCT comparison between the two groups. (c) TNF-*α* comparison between the two groups. ^#^means comparison with before intervention (*P* < 0.05), ^&^means comparison with RG (*P* < 0.05).

**Figure 3:** Comparison of mobility before and after an intervention. (a) FMAscore comparison between the two groups. (b) HHS score comparison between the two groups. (c) BI index comparison between the two groups. ^#^means comparison with before intervention (*P* < 0.05), ^&^means comparison with RG (*P* < 0.05).

**Figure 4:** Comparison of psychological states before and after an intervention. A)GCQscore comparison between the two groups. (B) SASscore comparison between the two groups. (C) SDSscorecomparison between the two groups. ^#^ means comparison with before intervention (*P* < 0.05), ^&^ means comparison with RG (*P* < 0.05).

**Table 1:** Univariate analysis of factors influencing the occurrence of LEDVT.

Factors	DVT group (*n* = 79)	No DVT group (*n* = 189)	*χ* ^2^	*P*
Age (year)			30.560	<0.001
<60	41 (51.90)	159 (84.13)		
≥60	38 (48.10)	30 (15.87)		

BMI (kg/m^2^)			9.927	0.002
<25	43 (54.43)	140 (74.07)		
≥25	36 (45.57)	49 (25.93)		

Gender			0.008	0.780
Male	42 (53.16)	104 (55.03)		
Female	37 (46.84)	85 (44.97)		

Limb paralysis			85.630	<0.001
Yes	56 (70.89)	26 (13.76)		
No	23 (29.11)	163 (86.24)		

Concomitant disease			9.263	0.026
Diabetes	22 (27.85)	69 (36.51)		
Hypertension	41 (51.90)	61 (32.28)		
Coronary heart disease	8 (10.13)	29 (15.34)		
None	8 (10.13)	30 (15.87)		

CVC of lower limbs			22.950	<0.001
Yes	41 (51.90)	42 (22.22)		
No	38 (48.10)	147 (77.78)		

Type of surgery			0.636	0.959
Brain surgery	8 (10.13)	16 (8.47)		
Thoracotomy	23 (29.11)	62 (32.80)		
Abdominal surgery	27 (34.18)	60 (31.75)		
Bone surgery	17 (21.52)	43 (22.75)		
Other	4 (5.06)	8 (4.23)		

Bedridden time (d)			17.070	<0.001
≤5	42 (53.16)	148 (78.31)		
>5	37 (46.84)	41 (21.69)		

**Table 2:** Assignment for multivariate analysis of factors.

Influencing factors	Assignment
Age (year)	<60 = 0, ≥60 = 1
BMI (kg/m^2^)	<25 = 0, ≥25 = 1
Limb paralysis	No = 0, Yes = 1
Combined hypertension	No = 0, Yes = 1
CVC of lower limbs	No = 0, Yes = 1
Bedridden time (d)	≤5 = 0, >5 = 1

**Table 3:** Multivariate analysis of factors affecting the occurrence of LEDVT.

Influencing factors	*B*	S.E.	Wald *χ*^2^	*P*	OR	95%CI
Age	0.892	0.742	1.445	0.637	2.440	0.569–10.447
BMI (kg/m^2^)	0.663	0.429	2.388	0.421	1.940	0.837–4.498
Limb paralysis	0.742	0.346	4.599	<0.001	2.100	1.065–4.137
Combined hypertension	0.701	0.340	4.251	<0.001	2.015	1.035–3.925
CVC of lower limbs	0.711	0.211	11.354	<0.001	2.036	1.346–3.078
Bedridden time	0.439	0.214	4.208	<0.001	1.551	1.019–2.359

**Table 4:** Comparison of satisfaction.

Group	Very satisfied	Basically satisfied	Dissatisfied	Overall satisfaction rate
RG (*n* = 36)	24 (66.67)	10 (27.78)	2 (5.56)	94.44%
CG (*n* = 43)	15 (34.88)	19 (44.19)	9 (20.93)	79.07%
*χ* ^2^				3.865
*P*				0.049

## Data Availability

The raw data supporting the conclusion of this article will be available by the corresponding author upon request.
